# Sensor Type, Axis, and Position-Based Fusion and Feature Selection for Multimodal Human Daily Activity Recognition in Wearable Body Sensor Networks

**DOI:** 10.1155/2020/7914649

**Published:** 2020-06-07

**Authors:** Abeer A. Badawi, Ahmad Al-Kabbany, Heba A. Shaban

**Affiliations:** ^1^Electronics and Communications Engineering Department, Arab Academy for Science, Technology & Maritime Transport (AASTMT), Alexandria, Egypt; ^2^Intelligent Systems Lab, Arab Academy for Science, Technology & Maritime Transport, Abu Kir Campus, Alexandria, Egypt; ^3^Department of Research and Development, VRapeutic, Cairo, Egypt

## Abstract

This research addresses the challenge of recognizing human daily activities using surface electromyography (sEMG) and wearable inertial sensors. Effective and efficient recognition in this context has emerged as a cornerstone in robust remote health monitoring systems, among other applications. We propose a novel pipeline that can attain state-of-the-art recognition accuracies on a recent-and-standard dataset—the Human Gait Database (HuGaDB). Using wearable gyroscopes, accelerometers, and electromyography sensors placed on the thigh, shin, and foot, we developed an approach that jointly performs sensor fusion and feature selection. Being done jointly, the proposed pipeline empowers the learned model to benefit from the interaction of features that might have been dropped otherwise. Using statistical and time-based features from heterogeneous signals of the aforementioned sensor types, our approach attains a mean accuracy of 99.8%, which is the highest accuracy on HuGaDB in the literature. This research underlines the potential of incorporating EMG signals especially when fusion and selection are done simultaneously. Meanwhile, it is valid even with simple off-the-shelf feature selection methods such the Sequential Feature Selection family of algorithms. Moreover, through extensive simulations, we show that the left thigh is a key placement for attaining high accuracies. With one inertial sensor on that single placement alone, we were able to achieve a mean accuracy of 98.4%. The presented in-depth comparative analysis shows the influence that every sensor type, position, and placement can have on the attained recognition accuracies—a tool that can facilitate the development of robust systems, customized to specific scenarios and real-life applications.

## 1. Introduction

Accurate and timely recognition of human daily activities, throughout the day, is required in remote health-monitoring and care-giving systems [1]. One approach for recognizing human activities is to analyze the biosignals acquired using on-body sensors, which has been addressed by a significant body of research to date [2]. This attention has been stimulated by several factors, including the advances in machine learning techniques. These techniques represent a powerful tool for figuring out patterns in the biosignals, with which they can be differentiated and thus recognized. The literature has witnessed several datasets which are constructed to facilitate effective and efficient model learning, with interdataset variations that include the number of subjects, the types of sensors, and the positions of sensors, in addition to others [3]. Efficient inference using the learned models has necessitated the identification of the most indicative features in the dataset. This can be done using feature selection techniques which have been used often to simplify the learned models, reduce the computational complexity in real-life applications, and enhance the recognition accuracies as well.

In this work, we employ the Human Gait Database (HuGaDB) [4]. This is a recently constructed dataset which has several unique characteristics for studying human activity recognition. It provides biosignals acquired using three of the most widely used types of sensors in the field, namely, gyroscopes, accelerometers, and electromyography (EMG) sensors, placed on the left and right feet, shins, and thighs. Another reason for choosing such a dataset is that it considers the most comprehensive set of activities in the literature (twelve activities). It covers daily static and dynamic activities which represent a rich source of information that empowers effective model learning and thus accurate recognition.

Our own previous research [5] investigates the relation between the recognition accuracy and the IMU's placements-and-orientations [5]. We also highlight the impact (in terms of accuracy) of applying feature selection techniques on the IMU's data [6]. This research, however, studies the fusion of EMG sensor data with the IMU's data. Particularly, we incorporate our knowledge on the best sensor placements-and-orientations, in addition to our findings on the impact of feature selection, and we show that EMG data can influence the system's recognition capacity positively. In this work, we have considered widely used classifiers, namely, support vector machine (SVM), naive Bayes (NB), neural networks as multilayer perceptron (MLP), decision tree (DT), *k*-nearest neighbor (*k*-NN), and random forest (RF) [5]. We have also followed the study in [6] while applying feature selection. Hence, we used the different approaches for sequential feature selection including sequential forward feature selection (SFS), sequential backward feature selection (SBS), and sequential forward floating feature selection (SFFS) [6].

The contributions of this research can be summarized as follows:

1. Identifying, for each sensor (accelerometer, gyroscope, and EMG), the direction and the sensor position that achieved the highest accuracies for human activity recognition, in addition to the best classifier from the six different algorithms applied
2. Demonstrating that using the best axis for a sensor, together with the best classifier and selected features, can lead to a competitive performance that is close to the performance achieved considering the whole three axes of that sensor
3. Showing that feature selection methods yield a significant improvement in the recognition accuracies, with an approximate of half the number of the original features retained
4. Attaining the highest recognition accuracy on HuGaDB using sensor fusion (of accelerometers, gyroscope, and EMG) and off-the-shelf feature selection technique

The rest of this article is structured as follows.  Section 2 highlights the literature review. A discussion on the used dataset and the methods used for data processing is provided in Section 3.  Section 4 gives numerical results. Finally, the conclusion is provided in Section 5.

## 2. Related Work

Wearable sensors, such as accelerometers and gyroscopes, are widely used for human activity recognition. Because accelerometers measure linear acceleration, they fail to identify actions that are characterized by (or involve) joint rotation. Hence, combining gyroscopes, which measure rotational motion, with accelerometers can overcome such a problem. These two sensors are normally integrated in one wearable inertial mobile unit (IMU).

Another type of wearable sensors is the surface electromyography (sEMG). The myoelectric signal measured by the sEMG represents the electrical current associated with muscular action; hence, it can play an important role in activity recognition. In this study, we consider wearable inertial sensors and sEMG sensors placed on different positions of the body. In addition, we consider other major aspects of comparison including the number of subjects, features, activities, sensor placements, and types, and finally the various types of classifiers (the machine learning algorithms) used.

Among the previous work on human activity recognition is the scheme presented in [7]. The study involved 10 participants, each performed 7 activities, and the signals were collected from accelerometers on the ankle and the wrist. Eleven features were extracted from the signals corresponding to each activity, and finally, *k*-NN and artificial neural networks were used as classifiers, which achieved an accuracy of 97%. In pursuit of the highest recognition accuracies, the authors of [8] investigated different classification techniques, such as SVM, regularized linear regression, and Adaboost. These methods were used to classify 7 different activities from 10 subjects, and 5 features were extracted from accelerometers placed on 3 different places on the body. Finally, the average accuracy for subject-independent, subject-adaptive, and subject-dependent accuracies was 78.2% from Adaboost.

A novel method was proposed for activity identification in [9], with 15 subjects and 3 sensors; 18 actions were performed, and accelerometers were used with 4 features extracted from the signal. Finally, a decision tree algorithm is used to classify the activities, and it attained a 93.8% accuracy.

In [10], the adopted setup involved accelerometers on 4 different body positions to recognize 5 activities, and 4 subjects participated in the study. The authors extracted 12 features, and 3 machine learning algorithms were used for classification. The accuracy was calculated per subject, and the average accuracy for the three subjects and one subject vs all is 81% using the HMM classifier.

In the context of activity classification, the performance on two datasets was compared in [11]. The first dataset used accelerometer readings from the chest during a walking activity from 18 subjects, with 9 features extracted. The reported average accuracy was 99.8% using random forest, just for the walking activity. The second dataset consisted of six activities from 30 subjects, collected using accelerometers and gyroscopes, where the signals were collected from the waist. The study included 10 classification algorithms that were applied on 24 features and attained an average accuracy per activity that equals to 99.9%.

Surface electromyography (sEMG) and accelerometer sensors were used for monitoring daily activities of stroke patients in [12]. The sEMG and accelerometer data were recorded from 10 patients while doing 11 activities. The data prediction stage of the proposed pipeline was done using a multilayered neural network. The author calculated the sensitivity and specificity. Hence, we used both of these figures to compute the accuracy, which reached 97.4%, in order to be able to compare it with the literature.

The research in [13] introduced MyoGym which included 8 electromyogram sensors and a 9-axis unit containing 3-axis gyroscope, 3-axis accelerometer, and 3-axis magnetometer. The data were collected from 10 subjects, performing 30 different gym activities. Linear discriminant analysis (LDA) and quadratic discriminant analysis (QDA) were used to classify the different activities. The accuracy for all sensors combined together was 71.6% using LDA.

Recently, a new method was proposed in [14] to recognize human activities based on a feature selection approach. The signals corresponding to 13 different activities were collected using accelerometers and gyroscopes from the ankle, wrist, hip, and chest. Nineteen different features were extracted and only k-NN was used for classification, and it attained 99.13% accuracy. Another method for dynamic segmentation of features was proposed in [15]. An accelerometer sensor placed on the wrist was used to predict 12 different activities from 10 subjects, and finally, 14 features were extracted for classification using the following methods: DT, SVM, *k*-NN, MLP, and NB, with 94.21% accuracy attained using SVM.

In [16], two datasets were used for activity recognition. The first dataset involved 31 subjects, and the second dataset involved 30 subjects. In both datasets, accelerometers and gyroscopes were located on the waist. Also, the participants performed 6 different activities, and 17 features were adopted. This research involved two classifiers, namely, SVM and RF, with 5 types of ensemble classifiers—Bagging, Rotation Forest, Adaboost, Random Subspace, and Ensembles of Nested Dichotomies. The highest accuracies attained were 95.33% using the SVM classifier for the first dataset and 99.22% for the second dataset. Finally, a literature review was released in 2018 for sensor-based datasets that were constructed for human activity recognition [3]. It reviews the various types of sensors and devices used in the literature. There are three datasets that are related to our research, namely, UCI-HAR dataset [17], Opportunity AR dataset [18], and mHEALTH [19].

In this research, we use 3 types of sensor data (accelerometer, gyroscope, and electromyography) and six classification techniques to classify the activities, in addition to four feature selection algorithms. Also, 12 activities and 7 different sensor placements, with 18 subjects, are considered. According to the literature survey presented earlier, and the summary in Table 1, this study has three merits:

1. It investigates the effectiveness of the electromyography sensor when it is combined with accelerometer and gyroscope sensors to recognize human activities
2. It presents a thorough comparison between the different types of commonly used machine learning techniques and feature selection methods, while at the same time, taking into consideration other aspects of comparison, such as the number of subjects and activities
3. It achieves a significantly high accuracy (99.8%) on a recent-and-comprehensive dataset

In Table 1, we summarize the most recent and pertinent work in the literature. The comparison includes studies that adopted accelerometers alone, or accelerometers with gyroscopes and electromyography. In our comparison, we also included the number of subjects, activities, features, sensor position, classification methods, and the average accuracy. We also show different performance metrics that were used by the pertinent literature in Table 2. It can also be seen from this table that accuracy is the most widely used metric in the literature.

## 3. Methodology

### 3.1. Dataset Description

The Human Gait Database (HuGaDB) by Roman Chereshnev is used in this work [4]. This dataset contains twelve activities, with the following ID numbers: walking with ID number [0], running with ID number [1], going down with ID number [2], going up with ID number [3], sitting with ID number [4], sitting down with ID number [5], standing up with ID number [6], standing with ID number [7], bicycling with ID number [8], down by elevator with ID number [9], up by elevator with ID number [10], and sitting in the car with ID number [11]. The data was collected from 18 adults (14 males and 4 females).

Six body inertial wearable sensors were located in the left and right shin, thigh, and foot with a total of six placements, for accelerometers and gyroscopes. Electromyography sensors were placed on vastus lateralis. The samples were collected from 3-axis accelerometer, 3-axis gyroscope, and surface electromyography (sEMG) sensors, which yield a total number of 38 signals, 36 signals from the inertial sensors and 2 signals from the sEMG sensor. In addition to being recent and well-documented, the choice to work on the HuGaDB dataset is inspired by the inertial nature of the sensors used to collect the signals. This enables us to study how the individual movements of the different parts of the two legs can help in predicting the human activity.

### 3.2. Data Preprocessing

Our proposed pipeline starts with a preprocessing stage which involves signal normalization and segmentation. Due to the difference in units and ranges of the collected data (from the 3 types of sensors), it was required to normalize it using zero-mean and unit variance as shown in the following equation:

(1) $$\begin{array}{c} f_{\text{norm}}=\frac{f_{\text{raw}}-\mu }{\sigma }, \end{array}$$

where *µ* and *σ* are the mean and standard deviation, respectively.

Following the literature, most of the activity classification methods use windowing techniques for dividing a time-series signal into smaller segments. In this work, we use time-based sliding windows with 50% data overlap [20]. This overlap percentage is commonly used for activity recognition and was shown to yield the highest recognition accuracies [21].

### 3.3. Feature Extraction and Selection

Accurate and efficient activity recognition requires the selection of the most relevant features and/or the removal of redundant information. The two steps of feature extraction and selection are meant to serve this purpose. In this research, we adopt the commonly used statistical and time domain-based features proposed in the literature for accurate human activity recognition (HAR) [22, 23].  Table 3 shows the features used, their definitions, and the signals from which we extracted those features [24–26].

Feature selection is commonly used for dimensionality reduction. In this research, we aim to investigate the impact of sequential feature selection (SFS) algorithms on the recognition accuracy. Particularly, we adopt the following feature selection methods: (1) sequential backward selection, (2) sequential forward selection, (3) sequential backward floating selection (SBFS), and (4) sequential forward floating selection (SFFS). The notable merit of the SFS family of algorithms is their simple implementation. Basically, this group of greedy algorithms sequentially adds one feature at a time and retains that feature if it yields a better classification accuracy [27]. SFFS and SBFS implement the forward and backward step at every iteration to ensure that the feature selected is the best with the previous and the next subset of features.

### 3.4. Classification Techniques

In this work, we recognize activities in the HuGaDB dataset using a set of well-studied machine learning techniques, namely, multilayer perceptron (MLP), naive Bayes (NB), random forest (RF), *k*-nearest neighbor (*k*-NN), support vector machine (SVM), and decision tree (DT). As was mentioned in Section 2, these techniques are widely used in the field of activity recognition from wearable sensors. The reported performance in this study is based on the accuracy and a 10-fold cross validation.

### 3.5. Signal-Processing Method

We elaborate below on the pipeline of the proposed system, which is composed of three stages. To justify each step, we show the impact it has on the ultimate recognition accuracies. Stage one aims to classify the activities from accelerometer and gyroscope sensors to find the best classifier and the most revealing sensor placement. Stage two is meant to highlight the effect of using feature selection. Finally, the last stage aims to investigate the fusion of the outputs of the three sensors, namely, accelerometer, gyroscope, and electromyography sensor.  Figure 1 shows the pipeline of the proposed method. We elaborate on it in the following points:

1. The dataset used in our research is collected from the thigh, foot, and shin for both left and right legs. Accelerometer and gyroscope signals contain (*x*, *y*, *z*) components. Their magnitude is also added as a feature.
2. Each sensor detects twelve different signals that correspond to the different activities from eighteen subjects.
3. Each signal is then normalized to have the same range for all sensors, and then a fixed-length window is applied to each signal with 100 samples and a 50% overlap.
4. Next, we extract 14 features from each window.
5. The optimal number of features is computed from the signals by applying the four different types of sequential feature selection to select the most important information. Each signal obtained different number of features to achieve the highest accuracy.
6. We divide the dataset to a 70–30 ratio for training and testing to apply the aforementioned six machine learning algorithms.
7. Fusion of sensors is then implemented between the accelerometer-and-gyroscope signals and the electromyography signal. Electromyography signal goes throw the same aforementioned steps before getting fused with other sensors.
8. Investigating the fusion between sensors is done according the three following approaches: (1) accelerometer and electromyography signals, (2) gyroscope and electromyography signals, and (3) accelerometer, gyroscope, and electromyography signals.

## 4. Results and Discussion

We dedicate this section to highlight the results attained by applying the machine learning classifiers that were discussed in Section 3, on the HuGaDB dataset. For simulations, the code was written in Python, and we used the Scikit-learn library for applying the different machine learning techniques. The 6 classification methods mentioned in Section 3 are applied on each axis and magnitude, position on the right and left legs, and the combination of the sensor parameters.  Table 4 indicates the parameters we used for each of the adopted classifiers. We also compare the performance achieved using three aforementioned sensors accelerometer, gyroscope, and electromyography sensor, and the accuracies obtained from the optimal system. The discussion of the results starts by focusing on accelerometers and gyroscopes, and later in this section, we expand the presentation to involve the sEMG sensor. Furthermore, we discuss the impact of applying the SFS family of feature selection techniques on the recognition accuracy of the proposed system.

### 4.1. Performance Evaluation for Optimal Sensor Placement

To evaluate the best sensor placement, we considered the accelerometer and gyroscope sensors only, because of their ability to recognize the activities accurately as mentioned in our previous work [5]. The classification techniques were applied on the dataset of the inertial sensor placements, axes, and magnitude, in addition to the EMG sensor. As the inertial sensors are placed in three different placements on both legs, the total number attributes is 24 per leg, i.e., a total of 48 attributes for the left and right legs.  Figure 2 depicts a boxplot for the accuracies of the left leg accelerometer (total of 24 attributes). The figure demonstrates that the highest accuracy attained from the different placements and orientations of left leg accelerometer is 90.7% using the random forest algorithm. This accuracy is obtained from the *x*-axis component of the accelerometer on the thigh. DT and SVM achieved 89.4% and 88.1%, respectively, on the accelerometer's data. The right leg showed almost similar accuracies. The results obtained in this section, with regards to the best sensor placement, will affect the rest of the pipeline as will be shown in the following sections after adding the EMG sensor to these best positions and axes.

### 4.2. Optimal Classifier and Feature Selection Algorithm

#### 4.2.1. Performance Evaluation for Optimal Classifier

First, we started by investigating the classification accuracies of the accelerometer and gyroscope sensors attained from the left leg. We compared between three different positions, namely, the foot (lf), the thigh (lt), and the shin (ls). The random forest (RF) has consistently outperformed the other classifiers, while the least effective classifiers are the *K*-NN and the naive Bayes. Although random forest, support vector machine, and decision tree classifiers have proven significant effectiveness, the RF classifier's interquartile range (IQR) shows superior consistency when varying the sensor positions compared to the other classifiers' IQR. Later in this discussion, we elaborate further on the superiority of the random forest classifier with regards to the consistency across varying sensor placements. It is worth mentioning that this aligns with other conclusions in the literature with regards to the superiority of the random forest classifier over other classifiers [5], followed by SVM and DT, and the same steps were repeated to observe the changes after the EMG sensor addition.  Figure 3 shows the confusion matrix of the RF classifier. The predicted label activities versus the true label showed only three wrong detections:

1. For ID 11 (sitting in the car), it was predicted as ID 6 (sitting) twice
2. For ID 7 (standing), it was predicted as ID 8 (cycling)
3. For ID 6 (sitting), it was predicted as ID 11 (sitting in the car)

The accuracy reached 98.6%, and this result was obtained from both types of sensors (accelerometers and gyroscopes) and by setting the random forest number of trees to 256 instead of 10 (10 is the default number of trees in Scikit-learn library).

#### 4.2.2. Optimal Number of Features

This section presents a method for obtaining the optimal number of features. This is done by using cross-validation and the sequential feature selection family of algorithms, in order to score different feature subsets, and then choose the best number of features that attain the highest accuracy. The curve in Figure 4 shows a random example of our method. We chose the *y*-axis of the gyroscope sensor, and the figure shows that the curve reaches the maximum accuracy when *N* = 8, where *N* is the number of features. At that value of *N*, the variability in the performance is the least; also, it is followed by a gradual and almost-monotonic decline in the performance. The sky-blue shade above and below the blue curve shows the changing in the cross-validation, one standard deviation above and below the accuracy score shown in the curve. Our insight is that the decline following *N* = 8 is due to adding noninformative features to the model learning process. After investigating the performance of four sequential feature selection approaches, sequential forward floating feature selection attained the highest accuracy while retaining the minimum number of features compared to other methods. Those steps were repeated for the EMG signal on both legs to obtain the optimal number of features.

### 4.3. Comparison between Single Axis vs Triple Axes and All Features vs Selected Features

After selecting the optimal number of features for the best position (thigh on the left leg), we compare the performance achieved using all proposed features and that obtained using the four types of sequential feature selection approaches (backward, forward, backward floating, and forward floating). In this experiment, we included the classifiers that achieved the highest recognition accuracies in the previous experiments, support vector machine, random forest, k-NN, and the one that attained the least accuracies (decision tree). The comparison highlights the best output we obtained in Sections 4.1 and 4.2:

1. The best axis, namely, the *x*-axis for the accelerometer sensor and the *y*-axis for gyroscope sensor, both obtained from the left thigh
2. The combination of the best axes (*x*, *y*, and *z* axes and their magnitude)

Table 5 shows the classification accuracies obtained by the classifiers, before using feature selection, on the following sensor placements: *x*-axis of accelerometer (A_lt_*x*), *y*-axis of gyroscope (G_lt_*y*), and their combination (A_lt_*x* and G_lt_*y*). It also shows the accuracies after combining all the axes and their magnitude (A, G_lt_*x*, *y*, *z*, and mag) of both sensors. Finally, the last column shows the total number of features used in each try.

As mentioned earlier [6] and boldfaced in Table 5, the best accuracy is achieved using the RF classifier. The best single axis achieved 94.7% with 28 features, and the combination of all parameters achieved 96.8% with 112 features.  Table 6 shows the same comparison with feature selection taken into consideration. Our experiments showed that sequential forward floating feature (SFFS) selection outperforms other feature selection techniques.  Table 6 shows that using feature selection leads to higher classification accuracy than that with all features obtaining 96.9% with 15 features selected from the single axis and 98.4% with 37 features selected from all parameters.

To conclude this part of the results, we showed that using feature selection, higher recognition accuracies can be attained with an average 50% reduction in the total number of features as mentioned in [6]. We adopted the four types of the sequential feature selection family of techniques, which outperformed all other approaches. The comparison between the performance achieved using sensor data from the single axis and triple axes demonstrated that the single axis can be used and still achieve high accuracies to detect the activities, even though there is an information gain from using the data of the three axes. Furthermore, a comparison between accuracies before and after using feature selection showed a significant performance enhancement after eliminating redundant or noninformative features. We build up on the previous conclusion by determining the most informative features and then applying the different classifiers on the data of the best sensor position and direction.

### 4.4. Investigating the Impact of Fusing the EMG Data with Accelerometers and Gyroscopes

Comparison between accelerometers, gyroscopes, and electromyography sensor data for activity recognition have not received significant research attention in the literature. Specifically, the use of EMG sensors for daily activity recognition placed at different positions of the body has not received much attention.  Figure 5 shows a comparison between the classification accuracies of the six investigated classifiers and three types of sensor data without sensor data-fusion. As can be seen, EMG signal's classification accuracies are too low when used alone. This justifies the reason for not being widely used for activity recognition. However, EMG signals are important for applications that require muscle activity monitoring such as tele-rehabilitation. Accordingly, we investigate the impact of fusing the data from these three sensors on the accuracy of activity recognition. This section will be divided as follows: First, we compare the output of using jointly the data from accelerometers and electromyography sensor data to that of using the gyroscopes and electromyography sensor data. Finally, we discuss the fusion of these three sensor data with regards to accuracy, single axis versus triple axes, and the number of features after sensor fusion.

#### 4.4.1. Accelerometer and Electromyography Sensor Data

Accelerometers measure the linear acceleration that is applied to a device on all three axes (*x*, *y*, and *z*), including the force of gravity. However, electromyography is the collective electric signal from the muscles, which is managed by the nervous system and is produced while muscles contract. For the joint consideration of accelerometers and EMG sensor data, we repeat the same steps followed to generate the results in Tables 5 and 6. We compare between the best single axis of the accelerometer (left thigh *x*-axis) with the electromyography signal on one side and all the parameters of the accelerometer (*x*, *y*, *z*, and magnitude (mag)) with the electromyography signal on the other side.

Based on the conclusion in the previous section, we add our feature selection technique to the pipeline, in order to observe the improvement of the accuracies when the number of redundant or the noninformative features get eliminated. In Tables 7 and 8, it is shown that the *x*-axis component of the accelerometer and electromyography (A_lt_*x* + EMG) achieve a 92.31% accuracy using 28 features. On the other hand, using sequential forward floating selection obtains a 94.52% accuracy with only 16 features. Adding all accelerometer parameters to the electromyography signal (A_lt_all and EMG), the accuracy reaches 97.31% versus 98.22% after using feature selection; the corresponding number of features were 70 and 30, respectively.

#### 4.4.2. Gyroscope and Electromyography Sensor Data

Gyroscope measures the rate of a device rotation in rad/sec around each of the three axes (*x*, *y*, and *z*). With the results discussed below, we observe the relation between gyroscopes and electromyography sensors in the context of their ability to detect the muscle behaviour in addition to the muscle rotation and direction. We also observe the impact of the joint usage of these two sensors with and without feature selection. Although gyroscope and electromyography signals did not perform perfect separately, their combination leads to significant results. As shown in Table 9, random forest obtains the highest accuracy. The combination of data from the gyroscope's best single axis (*y*-axis) and the electromyography sensor (G_lt_*y* + EMG) achieves a 93.11% accuracy with 28 features. Considering all the gyroscope parameters jointly with EMG (G_lt_all + EMG), though, leads to a 95.41% accuracy with 70 features. On the other hand, our best feature selection algorithm (SFFS) decreases the number of features to 18 features for the best single axis for the gyroscope with the electromyography signals and still attains a 94.91% accuracy. Adopting feature selection with all the gyroscope parameters in addition to electromyography, the corresponding accuracy reaches 97.6% with 32 features only as shown in Table 10.

#### 4.4.3. Accelerometer, Gyroscope, and Electromyography Sensor Data

Finally, we study the fusion of the data gathered from three types of sensor data, in order to investigate how the different features from these heterogeneous signals interact together. The major three comparisons highlighted in our discussion are the performance corresponding to data from single axis versus triple axes, the number of adopted features, and the optimal sensor fusion output. We present these comparisons in Tables 11 and 12.  Table 11 demonstrates the results of combining the data from the best single axis for accelerometer and gyroscope together with the electromyography signal (A_lt_*x* + *G*_lt_*y* + EMG). The joint usage of the previous features yields a recognition accuracy of 95.20% with 42 features. Furthermore, by considering all the accelerometer and the gyroscope parameters with the EMG (left thigh acc + gyro all + EMG), the accuracy reaches 98.50% with a total of 126 features.  Table 12 features the same comparison in Table 9 while applying sequential forward floating feature selection. An accuracy of 97.1% is attained with 24 features only from the data of the single best axis, while 99.8% accuracy is attained with a total of 45 features from the data of all axes plus their magnitude in addition to the EMG signal.  Table 13 and Table 14 highlight the influence of changing the adopted validation protocol on the attained accuracy before and after applying feature selection.

The results presented in this section are summarized in Figures 6 and 7, as they illustrate the relation between the accuracy and number of features. We highlight the most significant outputs in our work in these points:

1. The best single axis and position that yield the highest accuracy, for the accelerometer and the gyroscope
2. Fusion between electromyography, and accelerometer, and gyroscope best single axis
3. Accelerometer and gyroscope fusion with all parameters (*x*, *y*, *z*, and magnitude)
4. Fusion between electromyography with all accelerometer and gyroscope parameters

Significant results are obtained as shown in Figure 6, where the number of features has almost decreased to the half after using sequential forward floating feature selection.  Figure 7 also shows impressing results in the perspective of accuracy. As shown in both figures, decreasing the number of features leads to higher accuracies in all cases, and that occurs because the unnecessary information from the signal was removed automatically and only the informative features were kept to classify activates perfectly. Finally, Table 15 shows selected features after the fusion of the three sensor data; these features achieved an accuracy of 99.8% with the least number of features.

## 5. Conclusion

Towards accurate recognition of daily human activities, this paper proposed a novel approach that is based on sensor fusion and feature selection. Other than performing feature selection and sensor fusion consecutively, our pipeline learns a model that selects indicative features by jointly considering heterogeneous signals. These signals are acquired from electromyography and wearable inertial sensors on the thigh, foot, and shin. We believe that this approach enables constructive interaction between features that would have been dropped (during feature selection) otherwise. We attained a mean recognition accuracy of 99.8% on HuGaDB—the highest on this dataset—which provides signals from different sensor types (gyroscopes, accelerometers, and sEMG sensors), placements, and positions. Using off-the-shelf feature selection methods and time-based and statistical features, the presented joint fusion-selection approach had successfully realized the potential of sEMG sensors and incorporated them effectively to benefit the performance of the system. Moreover, towards the development of less obstructive systems, we highlighted the potential of the left thigh as a key sensor placement for attaining high recognition accuracies. A mean recognition accuracy of 98.4% was attained using only one inertial sensor on that single placement. Through extensive simulations and comparative analysis, we justified the impact of every stage in the proposed pipeline and showed the influence of various system parameters on the recognition accuracy. This research is envisaged to facilitate building robust systems that are tailored to specific scenarios and real-life applications.

## Figures and Tables

**Figure 1:** Scheme of the proposed system adopted in this research.

**Figure 2:** Boxplots of different classifiers' accuracies for data from accelerometer signals (please see text for more details).

**Figure 3:** Confusion matrix for the random forest classifier from the accelerometer and the gyroscope sensors placed on the left thigh [5].

**Figure 4:** Gyroscope *y*-axis performance when the number of features is varied [6].

**Figure 5:** Six classification algorithm accuracies when applied on the *x*-axis signal from the foot, thigh, and shin of the left leg accelerometer, gyroscope, and EMG.

**Figure 6:** Difference in the number of features before and after using feature selection and sensor fusion.

**Figure 7:** Difference in accuracies attained with and without feature selection as shown in Figure 6.

**Table 1:** Review of the different techniques from the literature that are most-related to the proposed research.

Study	No. of subjects	No. of activities	No. of features	No. of positions	Sensor position	Sensor type	Classifiers	Average of classification accuracy
[7]	10	7	11	2	Wrist and ankle	Accelerometer	PNN and K-PNN	96%
[8]	10	7	5	3	Hip, thigh, and ankle	Accelerometer	SVM, regularized LR, and Adaboost	78.2%
[9]	15	18	4	3	Wrist, waist, and thigh	Accelerometer	Decision tree	93.8%
[10]	4	5	12	4	Left thigh, right arm, ankle, and abdomen	Accelerometer	SVM, AMM, HNN	81% avg. per subject
[11]	30	6	24	1	Waist	Accelerometer and gyroscope	RF, SVM, NB, J48, NN, K-NN, Rpart, JRip, Bagging, and Adaboost	99.8% avg. per activity
[11]	18	1	9	1	Chest	Accelerometer	NB, SVM, RF, J48, NN, K-NN, Rpart, JRip, Bagging, and Adaboost	99.9% avg. per activity
[12]	10	11	8	8	Arms, thigh, waist, and chest	Accelerometer and electromyography	ANN	97.4%
[13]	10	30	12	1	Arm	Accelerometer, gyroscope, magnetometer, and electromyography	LDA and QDA	71.6%
[14]	19	13	19	4	Chest, ankle, hip, and wrist	Accelerometer and gyroscope	k-NN	99.13%
[15]	10	12	14	1	Wrist	Accelerometer	DT, SVM, k-NN, MLP, and NB	96.87%
[16]	30	6	17	1	Waist	Accelerometer and gyroscope	SVM and RF	99.22%
[16]	31	6	17	1	Waist	Accelerometer and gyroscope	SVM and RF	95.33%
[17]	30	6	5	1	Waist	Accelerometer and gyroscope	Multiple HMMs, MOT, and k-NN	92.6%
[18]	4	4	—	14	Upper body, leg, and hip	Inertial sensors and accelerometers	DL (NMF + SAE)	99.9%
[19]	10	12	—	3	Chest, right wrist, and left ankle	Accelerometer, ECG, gyroscope and magnetometer	Hierarchical classification method HCM	97.2%
Ours	18	12	14	7	Right and left thighs, right and left shins, and right and left feet and an EMG on the thigh	Accelerometer, gyroscope and EMG	Neural networks, naive Bayes, random forest, (k-NN), SVM, and decision trees	99.8%

**Table 2:** Review of the different performance metrics that were used with pertinent techniques in the literature.

Study	Accuracy (%)	*F*1-score	Precision	Recall	CV method	Sensitivity (%)	Specificity (%)
[7]	96	—	—	—	Leave-one-out (LOOCV)	—	—
[8]	78.2	—	—	—	10-fold CV	—	—
[9]	93.8	—	—	—	Leave-one-out (LOOCV)	—	—
[10]	81	—	—	—	Leave-one-out (LOOCV)	—	—
[11]	99.8	—	—	—	5-fold CV	100	100
[12]	97.4	—	—	—	—	95	99.7
[13]	71.6	—	—	—	—	—	—
[14]	99.13	Avg. of all activities 98.86%	Avg. of all activities 98.77%	Avg. of all activities 98.95%	Leave-one-out (LOOCV)	—	—
[15]	96.87	85.84%	—	—	10-fold CV	84.7	85.3
[16]	99.22	Avg. of all activities 99.23%	Avg. of all activities 99.23%	Avg. of all activities 99.23%	10-fold CV	—	—
[16]	95.33	Avg. of all activities 95.52%	Avg. of all activities 95.52%	Avg. of all activities 95.50%	10-fold CV	—	—
[17]	92.6	—	—	—	—	—	—
[18]	99.9	99.4%	99.4%	99.4%	Leave-one-out (LOOCV)	—	—
[19]	97.2	97.2%	97.2%	97.2%	—	—	—
Ours	99.8	99.3%	99.1%	99.4%	10-fold CV	99.4	99.1

**Table 3:** Definition of the features extracted in the proposed research.

Feature	Description
Standard deviation	Standard deviations of (*x*, *y*, *z*, magnitude) from accelerometer, gyroscope signals, and EMG signal
Standard deviation Auto-correlation	Auto-correlation of the standard deviations of (*x*, *y*, *z*, magnitude) from accelerometer, gyroscope signals, and EMG signal *Adopted function*: statsmodels.tsa.stattools.acf (*x*, unbiased = false, nlags = 40, qstat = false, fft = none, alpha = none, missing = “none”)
Standard deviation Auto-covariance	Auto-covariance of the standard deviations of (*x*, *y*, *z*, magnitude) from accelerometer, gyroscope signals and EMG signal *Adopted function*: statsmodels.tsa.stattools.acv (*x*, unbiased = false, nlags = 40, qstat = false, fft = none, alpha = none, missing = “none”)
Variance	Variance of (*x*, *y*, *z*, magnitude) from accelerometer, gyroscope signals, and EMG signal
Mean	Mean of (*x*, *y*, *z*, magnitude) from accelerometer, gyroscope signals, and EMG signal
Mean Auto-covariance	Auto-covariance of the mean values of (*x*, *y*, *z*, magnitude) from accelerometer, gyroscope signals, and EMG signal
Mean Auto-correlation	Auto-correlation of the mean values of (*x*, *y*, *z*, magnitude) from accelerometer, gyroscope signals, and EMG signal
Minimum	Minimum value of (*x*, *y*, *z*, magnitude) from accelerometer, gyroscope signals, and EMG signal
Maximum	Maximum value of (*x*, *y*, *z*, magnitude) from accelerometer, gyroscope signals, and EMG signal
Skewness	Asymmetry of (*x*, *y*, *z*, magnitude) from accelerometer, gyroscope signals, and EMG signal *Adopted function*: scipy.stats.skew (a, axis = 0, bias = true)
Kurtosis	Fourth central moment value divided by the variance square value of (*x*, *y*, *z*, magnitude) from accelerometer, gyroscope signals, and EMG signal *Adopted function*: scipy.stats.skew (a, axis = 0, bias = true)
Root-mean squared	Square root of the mean square (*x*, *y*, *z*, magnitude) from accelerometer, gyroscope signals, and EMG signal
Mean crossing rate	Mean crossing rate of (*x*, *y*, *z*, magnitude) from accelerometer, gyroscope signals, and EMG signal
Jitter	Jitter of (*x*, *y*, *z*, magnitude) from accelerometer, gyroscope signals, and EMG signal, where the jitter is defined as the deviation of a signal's significant instants from their ideal positions in time

**Table 4:** Parameters of each of the adopted classifiers.

Classifiers	Parameters
Multilayer Perceptrom	sklearn.neural_network.MLPClassifier(hidden_layer_sizes = (100,), activation = “relu”, solver = “adam”, alpha = 0.0001, batch_size = “auto,” learning_ate = “constant,” learning_rate_init = 0.001, power_t = 0.5, max_iter = 200, shuffle = True, random_state = None, tol = 0.001, verbose = False, warm_start = False, momentum = 0.9, nesterovs_momentum = True, early_stopping = False, validation_fraction = 0.1, beta_1 = 0.9, beta_2 = 0.999, epsilon = 1*e* ‒ 08, n_iter_no_change = 10, max_fun = 15000) We tested hidden_layer_sizes = (10, 20, 50, 75, 100) and hidden_layer_sizes = 100 gave best results

Decision tree (DT)	sklearn.tree.DecisionTreeClassifier(criterion = “gini,” spliter = “best,” max_depth = None, min_samples_split = 2, min_samples_leaf = 1, min_weight_fraction_leaf = 0.0, max_features = None, random_state = None, max_leaf_nodes = None, Min_impurity_decrease = 0.0, min_impurity_spilt = None, class_weight = None, presort = “deprecated.” ccp_alpha = 0.0)

Random forest (RF)	sklearn.ensemble.RandomForestClassifier(n_estimators = 128, criterion = “gini,” max_depth = None, min_samples_spilt = 2, min_samples_leaf = 1, min_weight_fraction_leaf = 0.0, max_features = “auto,” max_leaf_nodes = None, min_impurity_decrease = 0.0, min_impurity_split = None, bootstrap = True, oob_score = False, n_jobs = None, random_state = None, verbose = 0, warm_start = False, class_weight = None, ccp_alpha = 0.0, max_samples = None) We tested n_estimators = (10, 64, 12, 256), and n_estimators = 256 gave best results. Homwever, there was aslight difference compared to n_estimators = 128. So, we applied 128 to reduce the over all running time

k-Nearest neighbors (k-NN)	kNeighborsClassifier(n_neighbors = 5, weights = “uniform,” algorithm = “auto,” leaf_size = 30, p = 2, metric = “minkowski,” metric_params = None, n_jobs = None, ^*∗∗*^kwargs) We tested n_neighbors = (1, 5, 10, 20), and n_neighbors = 5 gave best results

Support vector machine (SVM)	sklearn.svm.SVC(C = 10, kernel = “linear,” degree = 3, gamma = “auto,” coef0 = 0.0, shrinking = True, probability = False, tol = 0.001, cache_size = 200, class_weight = None, verbose = False, max_iter = ‒1, decision_function_shape = “ovr,” break_ties = False, random_state = None We tested C = 1, 10, 20, 50, 100 and Kernel = “rbf” and “linear,” and the best results was obtained with gamma = “auto,” C = 10, and kernel = “linear”

Naive Bayes	sklearn.naive_bayes.GaussianNB (priors = None, var_smoothing = 1*e* ‒ 09)

**Table 5:** Comparison between accuracies attained using single axis and triple axes before using feature selection.

Sensor type and position	DT	SVM	RF	*k*-NN	Number of features
A_lt_*x*	88.10	89.40	90.70	79.10	14
G_lt_*y*	85.80	83.90	86.80	66.90	14
A_lt_*x* and G_lt_*y*	90.00	89.40	**94.70**	71.50	28
A, G_lt_*x*, *y*, *z* and mag	95.10	95.40	**96.80**	84.80	112

**Table 6:** Comparison between accuracies attained using single axis and triple axes after using feature selection.

Sensor type and position	DT	SVM	RF	*k*-NN	Number of features
A_lt_*x*	89.80	91.50	91.67	82.00	7
G_lt_*y*	88.10	85.20	88.70	87.80	8
A_lt_*x* and G_lt_*y*	91.60	91.20	**96.90**	75.00	15
A, G_lt_*x*, *y*, *z*, and mag	96.40	97.00	**98.40**	86.30	37

**Table 7:** Comparison between accuracies attained using single axis and triple axes for accelerometer and electromyography signals without using feature selection.

Sensor type and position	DT	SVM	RF	*k*-NN	Number of features
A_lt_*x*	88.10	89.40	90.70	79.10	14
EMG	76.90	78.90	79.20	66.20	14
A_lt_*x* + EMG	87.45	85.19	**92.31**	67.17	28
A_lt_all	92.03	93.60	95.00	83.90	56
A_lt_all + EMG	93.65	92.87	**97.13**	84	70

**Table 8:** Comparison between accuracies attained using single axis and triple axes for accelerometer and electromyography signals with sequential forward floating feature selection.

Sensor type and position	DT	SVM	RF	*k*-NN	Number of features
A_lt_*x*	89.80	91.50	91.67	82	7
EMG	78.00	80.30	84.30	70.10	11
A_lt_*x* + EMG	88.91	87.65	**94.52**	70.22	16
A_lt_all	94.20	95.10	96.20	85.10	23
A_lt_all + EMG	95.65	95.01	**98.22**	85.83	30

**Table 9:** Comparison between accuracies attained using single axis and triple axes for gyroscope and electromyography signals without using feature selection.

Sensor type and position	DT	SVM	RF	*k*-NN	Number of features
G_lt_*y*	85.80	83.90	86.80	66.90	14
EMG	76.90	78.90	79.20	66.20	14
G_lt_*y* + EMG	88.60	90.41	**93.11**	72.96	28
G_lt_all	87.90	88.60	92.50	81.20	56
G_lt_all + EMG	90.27	90.83	**95.41**	73.10	70

**Table 10:** Comparison between accuracies attained using single axis and triple axes for gyroscope and electromyography signals with sequential forward floating feature selection.

Sensor type and position	DT	SVM	RF	*k*-NN	Number of features
G_lt_*y*	88.10	85.20	88.70	87.80	8
EMG	78.00	80.30	84.30	70.10	11
G_lt_*y* + EMG	90.11	91.78	**94.91**	75.23	18
G_lt_all	89%	90.10	94.40	82.90	26
G_lt_all + EMG	93.13	92.83	**97.60**	76.32	32

**Table 11:** Comparison between single axis vs triple axes for accelerometer, gyroscope, and electromyography signals before using feature selection.

Sensor type and position	DT	SVM	RF	*k*-NN	No. of features
A_lt_*x*	88.10	89.40	90.70	79.10	14
G_lt_*y*	85.80	83.90	86.80	66.90	14
EMG	76.90	78.90	79.20	66.20	14
A_lt_*x* + G_lt_*y*	90.00	89.40	94.70	71.50	28
A_lt_*x* + G_lt_*y* + EMG	91.40	90.70	**95.20**	72.80	42
A_lt_all	92.03	93.60	95.00	83.90	56
G_lt_all	87.90	88.60	92.50	81.20	56
A, G_lt_all	95.10	95.40	96.80	84.80	112
A, G_lt_all + EMG	96.80	96.70	**98.50**	87.30	126

**Table 12:** Comparison between accuracies attained using single axis and triple axes for accelermoeter, gyroscope, and electromyography signals with sequential forward floating feature selection.

Sensor type and position	DT	SVM	RF	*k*-NN	No. of features
A_lt_*x*	89.80	91.50	91.67	82	7
G_lt_*y*	88.10	85.20	88.70	87.80	8
EMG	78.00	80.30	84.30	70.10	11
A_lt_*x* + G_lt_*y*	91.60	91.20	96.90	75.00	15
A_lt_*x* + G_lt_*y* + EMG	93.10	92.40	**97.10**	78.40	24
A_lt_all	94.20	95.10	96.20	85.10	23
G_lt_all	89	90.10	94.40	82.90	26
A, G_lt_all	96.40	97	98.40	86.30	37
A, G_lt_all + EMG	97.30	98	**99.80**	88.10	45

**Table 13:** Comparison between 10-fold CV and LOPO CV for accelerometer, gyroscope, and EMG sensors before applying feature selection.

Classifier/validation protocol	10-fold CV (%)	LOPO CV (%)
Random forest	98.5	98.9
SVM	96.7	96.5
Decision tree	96.8	96.3
KNN	87.3	86.8

**Table 14:** Comparison between 10-fold CV and LOPO CV for accelerometer, gyroscope, and EMG sensors after applying feature selection.

Classifier/validation protocol	10-fold CV (%)	LOPO CV (%)
Random forest	99.8	99.4
SVM	98	98.2
Decision tree	97.3	97.1
KNN	88.1	88.5

**Table 15:** List of input sources and the corresponding features acquired from them.

Input source	Features
A_lt_*x*	Jitter, mean, standard deviation, maximum, standard deviation auto covariance, standard deviation auto-correlation, and root-mean square
A_lt_*y*	Jitter, mean crossing rate, variance, minimum, maximum, standard deviation auto-correlation, kurtosis, and root-mean square
A_lt_*z*	Jitter, mean, standard deviation, minimum, variance, standard deviation auto covariance, skewness, and kurtosis
Ac_lt_mag	Mean and variance
G_lt_*x* G_lt_*y*	Mean, jitter, and standard deviation auto-correlation standard deviation, minimum, variance, mean auto correlation, root-mean square, and skewness
G_lt_*z*	Mean crossing rate, mean, mean auto covariance, and root-mean square
G_lt_mag	Mean crossing rate, standard deviation, standard deviation auto covariance, and root-mean square
EMG_l	Mean crossing rate, minimum, and kurtosis

## Data Availability

Previously reported wearable inertial sensor and EMG sensor data (HuGaDB) were used to support this study and are available at DOI: 10.1007/978-3-319-73013-4_12. These prior studies (and datasets) are cited at relevant places within the text as references [4].
